This article has been retracted.

# Prognostic influence of PD-1/PD-L1 suppressors in combination with chemotherapeutic agents for non-small cell pulmonary carcinoma: system review and meta-analysis

**DOI:** 10.3389/fonc.2023.1137913

**Published:** 2023-04-19

**Authors:** Min Shen, Chunxia Lu, Jie Gao

**Affiliations:** Department of Respiratory and critical care, Qidong People’s Hospital/Qidong Liver Cancer Institute/Affiliated Qidong Hospital of Nantong University, Qidong, China

**Keywords:** PD-1/PD-L1 inhibitors, chemotherapeutic drugs, NSCLC, short-term efficacy, prognosis

## Abstract

**Background:**

Lung cancer is a common malignant tumor, which is seriously harmful to human life and health. Nowadays, it has gradually become one of the best treatments for non-small cell lung cancer (NSCLC) to combine immunotherapy and chemotherapy, and its clinical efficacy is preliminary. Nevertheless, substantial differences exist between various studies and various indicators. Despite their unconvincing results, high-quality research evidence is needed to support them. In this case, further correlative studies are necessary to investigate the prognostic outcomes of PD-1/PD-L1 suppressors in combination with chemotherapeutic drugs in NSCLC.

**Methods:**

The online public databases were searchable for the clinical trials that consisted of NSCLC patients who had concluded their chemotherapy and who had accepted PD-1/PD-L1 suppressors. The time-span of the search spanned from the beginning to the end of the database. Two investigators retrieved the data independently. RevMan 5.3 statistical software was utilized for the assessment of bias risk. The software followed the Cochrane Handbook 5.3 guidelines.

**Results:**

There were seven clinically controlled studies with 2781 NSCLC samples finally included in this study. A meta-analysis of the post-treatment overall response rate (ORR) was undertaken. A remarkably higher ORR rate was observed in the study group (p<0.05). Study participants had a noticeably longer PFS (HR=0.61, 95% CI=0.54-0.70, P<0.00001). Study participants had markedly longer overall survival (OS) (HR=0.651, 95% CI=0.52-0.82, P<0.05). The incidence of adverse events (AEs) of Grade 3 or above was not clinically clearly different (P>0.05), as demonstrated by the incidence of AEs. The funnel plots were separately charted in accordance with ORR rate, PFE, OS, and Grade 3 AEs. The majority of the funnel plots were symmetrical and a minority of funnel plots were asymmetrical, indicating the heterogeneity of research and the limited evidence available may lead to some publication bias in the contained literature.

**Conclusion:**

The combined PD-1/PD-L1 inhibitors with conventional chemotherapy can dramatically elevate the prognosis of NSCLC patients, obviously enhancing the ORR rate and prolonging their PFS and OS. Furthermore, it was found that adding PD-1/PD-L1 inhibitors to conventional chemotherapy did not result in any additional adverse effects.

## 1 Background

Lung cancer is a common malignant tumor, which is seriously harmful to human life and health. In accordance with the latest research statistics of the International Agency for Research on Cancer (IARC) of the World Health Organization, there will be 82000 new cases of lung cancer in China happened in 2020, with 71000 deaths. Taking into account their histology, in addition to small cell lung cancer (SCLC), there is also non-small cell lung cancer (NSCLC), and the latter account for 85% of lung cancers (1). Surgical resection is the primary approach for the management of early-stage NSCLC currently. Nevertheless, the post-surgical patient prognosis and five-year survival remain dissatisfactory, with roughly two-thirds of patients with local or remote metastases by the time of detection (2). Typically, platinum-based chemotherapy is given to advanced NSCLC patients as their first course of treatment. Many patients cannot tolerate chemotherapy due to its pronounced side effects (3). The targeted therapies can be effective in controlling tumor growth in patients with particular genetic mutations and rearrangements. Many patients do not benefit from targeted therapy in the lack of driver mutations (4). Hence, novel therapeutic strategies and effective biomarkers for patients with NSCLC have emerged as a major direction to achieve improved patient prognosis.

Immune checkpoint inhibitor (ICI) drugs are capable of inhibiting the “off-work break-feed” signal by neoplastic cells (5), which can recover the proper immune system function and target tumor cells. At present, the major ICIs on the market are cytotoxic T-lymphocyte-associated antigen 4 (CTLA-4) suppressors and PD-1/PD-L1 suppressors, of which PD-1/PD-L1 suppressors consist of PD-1 antibodies and PD-L1 inhibitors (6, 7). ICI is widely recognized for its excellent efficacy and favorable safety profile for various tumors, which heralds a new era when treating malignant tumors. At present, four PD-1 inhibitors have been listed in China, namely Nivolumab (June, 2018), Pembrolizumab (July, 2018), Tislelizumab (December, 2018), and Sintilimab (December, 2018). Two PD-L1 inhibitors are listed in China, namely Durvalumab (December, 2019) and Atezolizumab (February, 2020). The Chinese government began 271 clinical trials in February 2021 involving PD-1/PD-L1 inhibitors, which are widely permitted for treating colorectal and lung cancers. According to a large number of clinical trials (8–10), the combination therapy has better OS and PFS when the tumor percentage score (TPS) of PDL-1 is ≥1% compared with PD-1/PD-L1 inhibitors alone. Nowadays, it has gradually become one of the best treatments for NSCLC to combine immunotherapy and chemotherapy, and its clinical efficacy is preliminary. Nevertheless, substantial differences exist between various studies and various indicators. Despite their unconvincing results, high-quality research evidence is needed to support them. In this case, further correlative studies are necessary.

## 2 Research contents and methods

### 2.1 Study design

The design was developed based on the preferred reporting items of the system review and meta-analysis plan. To comprehensively understand the effect of PD-1/PD-L1 inhibitor combined with chemotherapy drugs on the prognosis of non-small cell lung cancer through systematic review and meta-analysis.

### 2.2 Participants

All cases undergo pathological examination. The pathological type was NSCLC without EGFR, ALK and other driving gene mutations.

### 2.3 Interventions

PD-1/PD-L1 inhibitors (Pablizumab, Navumumab, Atrazumab, and Ipizumab) were administered along with standard chemotherapy to the study group, whereas standard chemotherapy or placebo was given to the control group.

### 2.4 Comparators

Compare the ORR, PFS and OS indicators of the included patients.

### 2.5 Systematic review protocol

#### 2.5.1 Literature inclusion criteria

(1) Study types: Clinical trials that did not involve PD-1/PD-L1 inhibitors and chemotherapy. Additionally, references were retroactively included in the literature to supplement and obtain relevant information. If the results of the same clinical control study were published in a series of articles, we contained only the latest and most comprehensive literature (2). Design type: clinical control study.

#### 2.5.2 Literature exclusion standard

(1) Clinical control studies were not conducted (2); As a result of the incomplete report, it was not possible to use the data (3); Recent studies were taken into consideration, and a repeat of the study’s content was conducted (4); there were no noticeable effects of the study in terms of curing. (5) studies that did not provide access to the full-text studies repeatedly published through multiple channels and studies in languages other than Chinese or English.

### 2.6 Search strategy and data source

Data about advanced NSCLC patients treated with PD-1/PD-L1-free inhibitors associated with chemotherapy were collected from PubMed, EMBASE, ScienceDirect, Cochrane Library, China National Knowledge Infrastructure (CNKI), VIP full-text (VIP), Wanfang Database and Chinese Biomedical Literature data (CBM), conference papers, degree papers. In addition to free words, subject words were searched, and key words included PD-1/PD-L1 inhibitors, chemotherapy, and patients with NSCLC; short-term efficacy; prognosis; meta-analysis; advanced prognosis from January 2010 to March 2022.

### 2.7 Study selection

The included references are imported into EndNote 20, and the repeatedly selected documents are eliminated through EndNote 20. Manual screening based on literature content. Next, two reviewers screen the study based on inclusion and exclusion criteria. The work of the two reviewers was carried out independently, and the reasons for the exclusion of the literature were recorded. The documents with differences are discussed by the third reviewer. The final step is to check whether there is any research overlap in all the included literature.

### 2.8 Data extraction

1) The study contained an assessment of bias risk. The bias risk estimate was performed with ReviewMan 5.4 based on Cochrane Handbook 5.3.
2) Literature screening and data extraction. A cross-check was conducted by two researchers on the results who conducted independent screenings of literature, gathered data, analyzed quality, and assessed quality. In case of lack of complete data in the literature, the authors of this paper would be contacted. Besides basic information about the authors, publication date and number of cases, the data extraction included information about interventions, therapeutic procedures and outcomes.

### 2.9 Statistical processing

RevMan5.3 software was derived from the Cochrane Collaboration Network Meta-analysis. Odds risk (OR) was adopted as an indicator, and the measured data were presented as mean difference (MD). Every effect quantity was calculated by using point estimates and 95% confidence intervals (CI). Heterogeneity was examined using χ 2 for heterogeneity and I2 was used to determine heterogeneity. If P>0.05 and I2<50%, it was considered homogeneous and the modified effect model was acquired for Meta-analysis; if P<0. 05 and I2≥50%, the combined effect was needed to determine homogeneity and a random-effects model was selected. During P<0.05, the original heterogeneities would not be chosen, descriptive analysis was applied. It was statistically remarkable that the differences existed (p<0.05). In addition, literature bias in publications was determined *via* inverted funnel plots. The asymmetry of the funnel plots was examined using Eggers’ test. For tests with P-values less than 0.1, we employed the Trimand Fill method to rectify for potential release bias.

## 3 Results

### 3.1 Results of literature retrieval and literature inclusion in general

Through computer database retrieval, 7 clinical controlled studies were finally contained (11–17), with a total of 2781 cases. In **Figure 1**, you can see a screening diagram, while in **Table 1** you can find basic characteristics of the articles.

**Figure 1:** illustration of literature screening. Records identified from*: Refers to a database of literature sources. Records excluded**: Refers to excluded documents.

**Table 1:** Basic characteristics of literature.

Include the literature	Year of publication	N	Intervention method		Outcome index	Research type	Grouping method	Blind or not
		(C/T)	C	T				
Jiang Y (11)	2021	42/42	CT	CT+ Pablizumab	234	Prospective study	Random number table method	No
Zhan QY (12)	2021	30/30	CT	CT+ Navuliu monoclonal antibody	234	Prospective study	Random number table method	No
Liu FY (13)	2021	42/42	CT	CT+ Navuliu monoclonal antibody	23	Prospective study	Random number table method	No
L Gandhi (14)	2018	202/405	CT+ Placebo	CT+ Pablizumab	124	Prospective study	Not specified	No
Lynch TJ (15)	2012	280/278	CT+ Placebo	CT+ Pablizumab	134	Prospective study	Not specified	No
West H (16)	2018	340/343	CT	CT+ Atezumab	134	Prospective study	Not specified	No
MA Socinski (17)	2019	232/473	CT	CT+ Atezumab	134	Prospective study	Not specified	No

C, control group; T, study group; ICIs, immunosuppressant; CT, chemotherapy; Palcebo; 1, Progression-free survival (PFS); 2:Overall response rate (ORR); 3:Overall survival (OS);4:Adverse reactions (AEs).

### 3.2 Study selection and characteristics

In this meta-analysis, all seven clinical controlled studies reported baseline patient status. A total of four studies didn’t describe the random method in detail and discussed detailed treatment measures that mentioned “random distribution” in the literature. It was found in the seven literature that there was a high number of blind methods as well as lost follow-up or withdrawals with detailed descriptions. The improved JADAD score of 7 articles was 3 or 4, all of which were of high quality. **Figures 2**, **3** illustrate the risk bias analysis.

**Figure 2:** Risk bias chart.

**Figure 3:** Summary chart of risk bias.

### 3.3 Synthesized findings

#### 3.3.1 Overall response rate

In this study, there were 7 clinical controlled studies with 2781 samples contained. The ORR rates after treatment were measured in a meta-analysis. Heterogeneity analysis results indicated that Chi^2^ = 0.83, df=2, P=0.66, I^2^ = 0%, indicating that a distinct heterogeneity could be observed in the study’s data. Using a fixed effect model analysis, study participants had a higher ORR rate (P<0.05, **Figure 4**). NSCLC patients with combined PD-1/PD-L1 inhibitor therapy on top of chemotherapy displayed the obvious growing of treatment efficacy.

**Figure 4:** Meta analysis forest map of CT+ICIs VS CT ORR rate.

### 3.3.2 Progression-free survival

On the basis of the PFS after treatment, a meta-analysis was conducted. The heterogeneity examination results indicated that Chi^2^ = 8.21, df=4, P=0.09, I^2^ = 51%, indicating that a distinct heterogeneity could be observed in the study’s data. Analyses of the data were based on the random effect model (**Figure 5**). PFS of the study group was noticeably longer (HR=0.61, 95%CI= 0.54-0.70, P<0.00001). This indicated that the combination of PD-1/PD-L1 inhibitor therapy based on chemotherapy could noticeably prolong the progression-free survival of patients with NSCLC.

**Figure 5:** Forest map of Meta analysis of PFS of CT+ICIs VS CT.

#### 3.3.4 Overall survival

The OS after treatment was analyzed in a meta-analysis. Heterogeneity analysis results indicated that Chi^2^ = 27.70, df=5, P<0.0001, I^2^ = 82%, indicating that a distinct heterogeneity could be observed in the study’s data. Based on the random effect model analysis, the study group had a noticeably longer OS (HR=0.651, 95%CI= 0.52-0.82, P<0.05). In combination with chemotherapy, PD-1/PD-L1 inhibitors noticeably extended the survival of patients with NSCLC (**Figure 6**).

**Figure 6:** Total lifetime of CT+ICIs VS CT (OS) Meta analysis forest map.

#### 3.3.5 Adverse effects

Clinically, AEs above Grade 3 required special intervention or face dose reduction or even drug withdrawal. Meta-analysis was conducted on AEs above Grade 3. Heterogeneity analysis results indicated that Chi^2^ = 23.26, df=6, P=0.0007, I^2^ = 74%. It indicated that a distinct heterogeneity could be observed in the study’s data. Using the random effect model, no noticeable differences were found in adverse reaction incidences (P>0.05, **Figure 7**). This suggested that the combination of PD-1/PD-L1 inhibitor therapy on the basis of chemotherapy did not noticeably increase the risk of AEs in NSCLC patients.

**Figure 7:** Meta analysis forest map of AEs above CT+ICIs VS CT level 3.

#### 3.3.6 Publication bias analysis

Funnel charts were drawn on the basis of ORR rate, PFE, OS and Grade 3 AEs respectively. The publication bias analysis was conducted (**Figures 8**–**11**). There were a few asymmetrical funnel charts among the results, but most were symmetrical, suggesting the study was heterogeneous and had a small sample size, resulting in publication bias in the literature.

**Figure 8:** Funnel chart based on ORR rate.

**Figure 9:** Funnel diagram based on PFS.

**Figure 10:** Funnel diagram based on OS.

**Figure 11:** Funnel chart based on level 3 and above Aes.

## 4 Discussion

Cancer-related deaths account for roughly 20% of all deaths caused by lung carcinoma, which represents one of the clearest malignancies (18). The incidence and mortality of lung carcinoma has dramatically risen globally. Lung cancer has no apparent signs and symptoms in the early stages, and approximately 2/3 of sufferers have an unresectable locally advanced or metastatic neoplasm at the initial diagnosis (19, 20). Only 15% of patients with advanced NSCLC survive 5 years after systemic therapy (21, 22). Over the past few years, first-line chemotherapy for patients with late-stage NSCLC has largely been dependent on a dual combination of platinum-based drugs and third-generation agents (23, 24). Chemotherapy is prone to complications, such as severe gastrointestinal symptoms and myelosuppression. Chemotherapy cannot result in a remarkable enhancement of patient survival and patients’ quality of life is seriously influenced (25, 26). Thus, it is urgent to find a more effective treatment method.

Immunotherapy is by far of the most promising strategies (27). Agents targeting ICIS, especially PD-1 and PD-L1 antibodies, and PD-1/PD-L1 inhibitors can potentially regulate the immune responses by preventing the interactions among PD-L1-expressing neoplastic cells and PD-1-expressing T cells (18, 28, 29), recovering the proliferation and activation of CD4+T/CD8+ cells, and thus suppressing the escape, proliferation, and metastasis of neoplastic cells (1, 30). The FDA has already authorized many PD-1/PD-L1 blockers for the second-line and first-line management of NSCLC. When PD-1/PD-L1 blockers are used to treat locally advanced or metastatic NSCLC, the clinical outcome has been dramatically enhanced (31, 32). In the clinical trial by Masuda T et al, the first-line therapy with pembrolizumab in advanced PD-L1 high expression NSCLC was linked with a 40% lower risk of death and markedly improved PFS (10.3%) in comparison to platinum-containing chemotherapy (33). In the MajemMclinical trial, atezolizumab has also demonstrated superior efficacy over chemotherapy (34). The clinical study by Reck et al. indicated that pembrolicumab as a single agent had remarkably better PFS and OS than platinum-based dual chemotherapy if the expression of PD-L1 was equal to or above 50% (35).

It is noteworthy that NSCLC patients can have a better survival time after ICI treatment, but some patients still fail to benefit. Additionally, NSCLC patients receiving ICI also experience immune-related adverse effects that are associated with improved survival. It was found that ICI combined with chemotherapy has good OS and PFS, and the treatment effect is better than ICI alone. PD-1/PD-L1 inhibitors are better controlled by glucocorticoid therapy even if adverse reactions can occur, and have a better prospect of application (36).

In the present study, 2781 cases were sampled from seven controlled clinical trials. In the study group, there was a marked improvement in ORR, indicating that chemotherapy combined with PD-1/PD-L1 inhibitors can remarkably enhance the efficiency of patients with NSCLC with remarkable short-term effects. PD-1 is a human immunoglobulin that specially binds to human PD-1, allowing PD-1 to interact with PD-L1 and PD-L2 ligands. In addition to achieving desirable therapeutic effects, it has outstanding clinical advantages as a targeted cancer treatment agent. Through the employment of PD-1/PD-L1 inhibitors in combination with conventional chemotherapy, further improvements in clinical outcomes can be achieved. In the meta-analysis, PFS and OS were remarkably prolonged after treatment in the study group. Combined treatment with PD-1/PD-L1 inhibitors on top of chemotherapy remarkably prolonged progression-free survival and OS in NSCLC patients and could remarkably improve the long-term prognosis of patients. Chemotherapy combined with PD-1/PD-L1 inhibitors promotes remarkable antitumor effects and prolongs patients’ survival.

Clinical management of AEs associated with combination chemotherapy with PD-1/PD-L1 inhibitors has proven to be an essential aspect of therapy (37, 38). The majority of adverse reactions in the combination therapy group can be relieved or disappeared with appropriate symptomatic treatment. In the combination therapy group, there was a relatively high incidence of Grade 3-5 colectasis and hepatitis, compared to the chemotherapy group, and most AEs could be controlled by withdrawal of drugs and other treatments. An analysis of the incidence of AEs after treatment was conducted. In terms of adverse reaction incidence, no significant differences were found. Patients with NSCLC cured with chemotherapy containing PD-1/PD-L1 inhibitors did not experience a dramatic increase in the risk of three or more AEs, suggesting they are safe. In addition, separate funnel plots were drawn based on ORR rate, PFE, OS, and Grade 3 AEs. In the included literature, most funnel plots were symmetrical and a few were asymmetrical. Studies of heterogeneity and a limited amount of literature can explain this, given the heterogeneity and limited amount of literature. The limitations of this study mainly contain few RCTs included in the studies and some heterogeneity between studies. Also, some studies did not limit or analyze baseline characteristics of patients, such as gender, age, race, and smoking status. A subgroup analysis was not possible because there were no data across trials to determine the source of heterogeneity. Follow-up studies are needed to confirm PD-1/PD-L1 inhibitors’ clinical effectiveness when linked with chemotherapy in patients with NSCLC.

## 5 Conclusion

When combined with conventional chemotherapy, PD-1/PD-L1 inhibitors can noticeably enhance the outcome of NSCLC patients, noticeably increasing the ORR rate and prolonging their PFS and OS. Furthermore, a combination of PD-1/PD-L1 inhibitors and conventional chemotherapy did not appear to increase AEs.

## Data availability statement

The datasets used and/or analysed during the current study are available from the corresponding author on reasonable request.

## Author contributions

MS were major contributors in writing the manuscript. CL collected the patient data. JG did literature searches, and revised the manuscript. All authors contributed to the article and approved the submitted version.
